# Construction of Training Program for Specialized Nurses in the Central Sterile Supply Department (CSSD) Based on Post Competency

This article has been retracted.

**DOI:** 10.1155/2022/3282245

**Published:** 2022-06-14

**Authors:** Zhaohui Song, Yuanhua Qin, Bei Huang, Zhihong Zhang

**Affiliations:** ^1^Liuzhou People's Hospital, Liuzhou, China; ^2^Liuzhou Traditional Chinese Medical Hospital, Liuzhou, China

## Abstract

**Objective:**

The aim of this study is to analyze the construction of a training program for specialized nurses in disinfection supply center (CSSD) based on post competency.

**Methods:**

Based on the theory of post competency, literature analysis, investigation, and expert consultation are used to establish training contents and methods.

**Results:**

Two rounds of expert consultation were conducted in this study. In the first round of expert consultation, 22 questionnaires were sent out and 21 valid questionnaires were received with an effective recovery of 95.45%. Seven experts (31.82%) proposed 53 suggestions for modification. A total of 21 questionnaires were sent out in the second round of expert consultation and 21 were effectively received with an effective recovery rate of 100.00%. In the first round of expert consultation, the mean importance score of 63 third-level indicators was 4.00–5.00 points, the standard deviation was 0.00–1.00, and the full score rate was 46.54%–100.00%. In the second round of expert consultation, the mean importance score of 67 third-level indicators was 4.05∼5.00 points, the standard deviation was 0.00–0.88, and the full score rate was 20.00%∼100.00%. In the first round of expert consultation, the Kendall coordination coefficient was 0.187. In the second round of expert consultation, the Kendall coordination coefficient was 0.2196, and the differences were statistically significant after *χ*^2^ test (*P* < 0.05). The coefficient of variation of each index in the second round of expert consultation ranged from 0.00 to 0.21.

**Conclusion:**

The CSSD-specialized nurse training program based on job competency constructed in this study takes job competency as the theoretical basis and uses a literature analysis method, survey research method, and expert consultation method to establish the content and method of training, the above methods are scientific and reasonable, and experts are motivated. It is highly authoritative, and the consultation opinions of experts at all levels of indicators tend to be consistent, which can provide reference for the training of CSSD specialized nurses.

## 1. Introduction

Central sterile supply department (CSSD) is the unit in the hospital that is responsible for the cleaning, sterilization, and supply of sterile medical instruments, instruments, and articles that are reused in various departments [1]. It is the key to participate in the prevention and control of nosocomial infection in hospitals to collect, clean, disinfect, sterilize, and supply all the medical instruments, instruments, and articles that need to be disinfected or sterilized and reused in hospitals through centralized management, so as to ensure the safety of patients [2]. Competency refers to the traditional intelligence test, knowledge, skills, and academic ability test. Competency can not accurately predict the performance or life success of complex jobs and high-level positions. The main characteristics of competence are personal attitude, values, self-image, motivation, and characteristics [3]. Post competency refers to the sum total of knowledge, skills, abilities and characteristics that enable employees to be competent for their posts and produce excellent work performance in their posts in a specific organization [4, 5]. Job competency-based training is based on training objects and key competencies required for specific positions, focusing on the characteristics of high performers that are more outstanding than ordinary performers, and developing more targeted training courses, so as to achieve better training results [6]. In 2012, the guidance on the implementation of hospital nurse post-management issued by the Ministry of Health clearly pointed out that nurse training should be demand-oriented and centered on post competency, highlight professional connotation, pay attention to practical ability improve humanistic literacy, and meet the needs of clinical nursing development [7, 8]. In this study, the competency-based CSSD specialized nurses training is based on the key competency characteristics required by the CSSD specialized nurse post. The training program (training methods and contents) is designed based on the key competency characteristics required by the CSSD specialist nurse post, and the key contents of the training are highlighted in a targeted manner, so as to achieve good training results.

## 2. Materials and Methods

### 2.1. Setup a Research Group

The research group consists of five members, including 1 director nurse, two deputy director nurses, one supervisor nurse, and one nurse. Group members are responsible for retrieving and analyzing literature, compiling expert consultation questionnaire, selecting expert consultation questionnaire, issuing expert consultation questionnaire, and data statistics and analysis.

### 2.2. Compile the Expert Consultation Questionnaire

Based on the theory of job competency, this study preliminarily compiled expert consultation questionnaire on the basis of literature analysis and research group discussion. The expert consultation questionnaire consists of four parts:

① Instructions.
② Questionnaire for general information of experts.
③ Experts used the Likert 5-level scoring method to evaluate the importance degree of indicators at all levels, with 5 being very important, 4 being relatively important, 3 being generally important, 2 being not too important, and 1 being not important. In view of the importance of indicators at all levels, index setting and school hour arrangement is reasonable to solicit expert opinions and suggestions. We take this as the basis for assessing the importance of various indicators.
④ The judgment basis table for the importance of indicators selected by experts and the judgment table for the experts' familiarity with the contents filled in the form [9].

### 2.3. Choose a Consulting Expert

Inclusion criteria for consulting experts are as follows:

① Have more than 10 years of experience in tumor clinical nursing and CSSD work in grade 3A hospitals or CSSD teaching work in universities.
② Bachelor degree or above, title of deputy chief physician or above, or head nurse;
③ Have a good understanding of the research content;
④ Informed consent and active participation. 22 experts were selected for two rounds of expert consultation.

### 2.4. Expert Advice

Experts were consulted by e-mail and a paper questionnaire [10]. After the first round of expert consultation questionnaires were collected, the researchers followed the principle of index screening (mean significance ≥3.5 points, coefficient of variation ≤0.25). The second round of the expert consultation questionnaire was formed by sorting out and analyzing the results of expert consultation, revising the corresponding indicators according to the modification opinions and suggestions of experts and the discussion opinions of the research group.

### 2.5. Statistical Method

Excel and SPSS21.0 were used for data statistics and analysis. The general data of experts were described by frequency, mean ± standard deviation (*x* ± *s*), and composition ratio. The positive degree of experts was expressed by the questionnaire recovery rate and efficiency. The degree of expert authority is expressed by authority coefficient. The degree of concentration of experts' opinions was expressed by the mean, standard deviation, and full score ratio of the importance score of each index.

## 3. Results

### 3.1. General Information of Experts

The general information of experts is shown in Table 1:

### 3.2. Expert Activeness

Two rounds of expert consultation were conducted in this study. In the first round of expert consultation, 22 questionnaires were sent out and 21 valid questionnaires were received with an effective recovery rate of 95.45%. Seven experts (31.82%) proposed 53 suggestions for modification. A total of 21 questionnaires were sent out in the second round of expert consultation and 21 were effectively received with an effective recovery rate of 100.00%.

### 3.3. Degree of Expert Authority

The authority coefficient of the experts in the two rounds was 0.89, the judgment basis of the index was 0.91, and the experts' familiarity with the index was 0.87.

### 3.4. Degree of Concentration of Expert Opinions

In the first round of expert consultation, the mean importance score of 63 third-level indicators was 4.00–5.00 points, the standard deviation was 0.00–1.00, and the full score rate was 46.54%–100.00%. In the second round of expert consultation, the mean importance score of 67 third-level indicators was 4.05–5.00 points, the standard deviation was 0.00∼0.88, and the full score rate was 20.00%–100.00%.

### 3.5. Degree of Coordination of Expert Opinions

In the first round of expert consultation, the Kendall coordination coefficient was 0.187. In the second round of expert consultation, the Kendall coordination coefficient was 0.2196, and the differences were statistically significant after *χ*^2^ test (*P* < 0.05). The coefficient of variation of each index in the second round of expert consultation ranged from 0.00 to 0.21.

### 3.6. CSSD Specialist Nurse Training Program Based on Post Competency

#### 3.6.1. Course Content

Through two rounds of expert consultation, the curriculum content of CSSD specialist nurses was revised as follows according to the principle of indicator selection, expert consultation opinions, and discussion among members of the research group:

① The first-level indicator “job competency” was refined into four core elements of job competency, namely, knowledge, skills, ability, and characteristics.
② The second-level indicators were adjusted according to the refinement of the first-level indicators, and two indicators, professional development ability and management ability, were added.
③ The third-level indicators were adjusted according to the determination of the second-level indicators, and finally, 4 first-level indicators, 11 second-level indicators, and 44 third-level indicators were formed. The first-level and second-level indicators are shown in Table 2:

The three-level indicators are shown in Table 3:

#### 3.6.2. Training Methods

The training methods used in this study include teaching form, learning form, inspection form, and effect evaluation. “Clinical practice for 3 months” is changed to “clinical practice lasted for 1 month”. A secondary index of implementation effect evaluation is added. The total period of theoretical training was revised from 50 to 42. Training methods for specialist nurses in disinfection supply centers based on post competency are shown in Table 4:

Two rounds of expert consultation were conducted in this study. In the first round of expert consultation, 22 questionnaires were sent out and 21 valid questionnaires were received with an effective recovery of 95.45%. Seven experts (31.82%) proposed 53 suggestions for modification. A total of 21 questionnaires were sent out in the second round of expert consultation and 21 were effectively received with an effective recovery rate of 100.00%. In the first round of expert consultation, the mean importance score of 63 third-level indicators was 4.00–5.00 points, the standard deviation was 0.00–1.00, and the full score rate was 46.54%–100.00%. In the second round of expert consultation, the mean importance score of 67 third-level indicators was 4.05–5.00 points, the standard deviation was 0.00–0.88, and the full score rate was 20.00%–100.00%. In the first round of expert consultation, the Kendall coordination coefficient was 0.187; In the second round of expert consultation, the Kendall coordination coefficient was 0.2196, and the differences were statistically significant after *χ*^2^ test (*P* < 0.05). The coefficient of variation of each index in the second round of expert consultation ranged from 0.00 to 0.21.

## 4. Discussion

Compared with the particularity of clinical work and the difference of personnel structure, nursing professional training in disinfection supply centers in China started late and is still in the stage of exploration and development [11, 12]. To build a good CSSD specialist, a nurse requires the improvement of comprehensive quality. This training focuses on the training of comprehensive ability of specialized nurses in the design of the course. In addition to the training of laws, regulations, and theoretical knowledge related to the disinfection supply center, quality education, scientific research ability, and management courses are added to the training course [13, 14], such as responsibility, executive ability, teamwork, communication skills, service marketing, and other courses [15]. At present, the current situation of the CSSD is where a nurse and workers exist at the same time, there is no fixed position responsibilities, division of labor is not clear, it is also as an independent professional, disinfection supply center without reason of national health nurses, because in recent years along with the specification of compulsory execution, disinfection supply center is still in its stage of development [16]. According to the specific situation of each region, the training of specialized nurses plays an important role in expanding the service scope of disinfection supply centers, ensuring the quality of work, improving the specialized skill level of disinfection supply centers, and promoting the development of specialized undertakings [17–19].

## 5. Conclusion

In conclusion, the CSSD-specialized nurse training program based on job competency constructed in this study takes job competency as the theoretical basis and uses a literature analysis method, survey research method, and expert consultation method to establish the content and method of training, the method selected in this study is scientific, and experts are motivated. It is highly authoritative, and the consultation opinions of experts at all levels of indicators tend to be consistent. Important indicators in the training content include the following:

① Basic knowledge of occupational protection.
② Cleaning and disinfection equipment program.
③ Packing quality inspection.
④ Critical thinking ability.
⑤ The sense of responsibility.

Important indicators of training methods include the following:

① Case seminar.
② Self-study.
③ Theoretical examination.
④ Carry out teaching and training.

which can provide reference and reference for the training of CSSD-specialized nurses.

## Figures and Tables

**Table 1:** General information of experts.

General information		Score
Cases		22
Gender	Male	7
	Female	15
Age (average)		43.52 ± 6.41
Education background	Bachelor	9
	Master	11
	Doctor	2
Title	Senior title	4
	Associate senior title	10
	Head nurse	8
Years of work in related field (average)		21.58 ± 9.57

**Table 2:** First-level and second-level indicators.

Indicators	Importance score	Coefficient of variation	Full score rate (%)
1 Knowledge	4.58 ± 0.25	0.08	81.25
1.1 Professional knowledge	4.57 ± 0.42	0.14	62.47
1.2 Knowledge of ethics and law	4.63 ± 0.17	0.06	96.54
1.3 Symptom assessment and management	4.47 ± 0.48	0.12	58.97
2 Skills	4.95 ± 0.02	0.01	98.52
2.1 Daily management	4.65 ± 0.27	0.05	85.14
2.2 Main support	4.77 ± 0.14	0.02	98.27
2.3 Equipment use and maintenance	4.56 ± 0.38	0.07	65.45
3 Ability	4.77 ± 0.09	0.08	81.26
3.1 Communication ability	4.92 ± 0.04	0.01	95.47
3.2 Professional development ability	4.36 ± 0.14	0.11	46.52
3.3 Management ability	4.85 ± 0.08	0.07	85.63
4 Trait	4.92 ± 0.04	0.05	92.28
4.1 Personal professional quality	7.58 ± 0.35	0.04	93.19
4.2 Cooperative spirit of group	4.67 ± 0.29	0.06	85.67

**Table 3:** Three-level indicators.

Indicators	Importance score	Coefficient of variation	Full score rate (%)
1.1.1 Basic knowledge of disinfection and sterilization	4.64 ± 0.36	0.08	69.54
1.1.2 Standard preventive knowledge	4.74 ± 0.26	0.07	57.14
1.1.3 Basic knowledge of occupational protection	4.61 ± 0.51	0.11	82.32
1.1.4 Nosocomial infection prevention and control requirements	4.27 ± 0.61	0.15	81.14
1.2.1 Basic knowledge of medical devices	4.26 ± 0.58	0.14	68.27
1.2.2 Classification of medical cleaning agents	4.39 ± 0.58	0.12	77.15
1.2.3 Standard for use of packaging materials	4.28 ± 0.48	0.11	81.22
1.2.4 Disinfection and sterilization monitoring standards	4.55 ± 0.47	0.10	45.58
1.3.1 Water and steam quality requirements	4.08 ± 0.59	0.08	66.78
1.3.2 Cleaning and disinfection equipment program	4.17 ± 0.62	0.12	95.24
1.3.3 working principle and parameters of sterilization equipment	457 ± 0.52	0.14	72.14
2.1.1 Occupational protection measures	4.59 ± 0.14	0.09	53.57
2.1.2 Occupational exposure treatment procedures	4.63 ± 0.14	0.12	76.32
2.1.3 Pretreatment	4.25 ± 0.47	0.08	77.25
2.1.4 Recycling	4.49 ± 0.32	0.07	74.12
2.1.5 Manual cleaning	4.81 ± 0.07	0.07	85.63
2.1.6 Mechanical cleaning	4.52 ± 0.14	0.15	84.17
2.2.1 Packing quality inspection	4.96 ± 0.04	0.04	86.32
2.2.2 To be loaded with sterilized items	4.25 ± 0.63	0.06	85.21
2.2.3 Unqualified sterilized articles	4.17 ± 0.07	0.08	84.39
2.2.4 Evaluate the effect of sterilization	4.36 ± 0.57	0.09	79.32
2.3.1 Use and maintenance of soft water and pure water equipment	4.39 ± 0.12	0.11	80.24
2.3.2 Use and maintenance of cleaning and disinfection equipment	4.57 ± 0.25	0.12	85.36
2.3.3 Use and maintenance of drying equipment	4.66 ± 0.14	0.13	84.12
2.3.4 Use and maintenance of medical sealing machine	4.52 ± 0.17	0.09	73.14
2.3.5 Use and maintenance of high temperature sterilization equipment	4.36 ± 0.24	0.11	75.98
2.3.6 Use and maintenance of low temperature sterilization equipment	4.77 ± 0.25	0.08	77.14
2.3.7 Emergency plan and processing process	4.39 ± 0.81	0.12	75.63
3.1.1 Communication and coordination skills	4.24 ± 0.38	0.11	82.62
3.1.2 Critical thinking ability	3.99 ± 0.58	0.16	85.26
3.2.1 Career planning ability	4.12 ± 0.64	0.14	85.29
3.2.2 Nursing research capability	4.65 ± 0.48	0.12	76.22
3.2.3 Teaching and training ability	4.14 ± 0.48	0.09	74.19
3.2.4 Autonomous learning ability	4.55 ± 0.25	0.14	75.26
3.3.1 Risk prevention capability	4.58 ± 0.69	0.13	77.25
3.3.2 Job management ability	4.14 ± 0.24	0.12	78.36
3.3.3 Emergency response capability	4.62 ± 0.36	0.14	79.14
4.1.1 Physical quality	4.21 ± 0.69	0.15	85.64
4.1.2 The sense of responsibility	4.59 ± 0.41	0.11	92.14
4.1.3 Active service consciousness	4.84 ± 0.01	0.05	93.25
4.1.4 Self emotion management	4.67 ± 0.36	0.04	91.57
4.2.1 Team cooperation	4.62 ± 0.34	0.10	65.39
4.2.2 Professional identity	4.44 ± 0.58	0.13	85.53
4.2.3 Interpersonal relationships	4.37 ± 0.51	0.12	85.74

**Table 4:** Training methods for specialist nurses in disinfection supply centers based on post competency.

Training methods	Classification	Importance score	Coefficient of variation	Full score rate (%)
Teaching form	Group discussion	4.52 ± 0.36	0.08	81.25
	Lecture	4.86 ± 0.24	0.09	85.55
	Situational drilling	4.58 ± 0.29	0.06	85.14
	Case seminar	4.96 ± 0.14	0.06	86.28
	Practice sharing	4.88 ± 0.32	0.08	80.23
	Clinical practice lasted for 1 month	4.78 ± 0.14	0.09	81.14

Learn form	Online learning	4.62 ± 0.48	0.09	61.28
	Collective teaching	4.38 ± 0.05	0.12	45.57
	Self-study	4.62 ± 0.38	0.11	72.21

Inspection form	Operation assessment	4.58 ± 0.52	0.13	66.58
	Theoretical examination	4.85 ± 0.35	0.08	81.14
	Dynamic evaluation	4.66 ± 0.51	0.12	72.26
	Graduation reply	4.39 ± 0.37	0.07	65.57

Effect evaluation	Complete case	4.86 ± 0.24	0.06	85.59
	Research papers	4.16 ± 0.78	0.17	47.95
	Follow-up implementation	4.52 ± 0.48	0.10	53.69
	Carry out teaching and training	4.59 ± 0.44	0.12	61.27

## Data Availability

The datasets used during the present study are available from the corresponding author upon reasonable request.
